# Epithelial-Mesenchymal Transition Markers and HER3 Expression Are Predictors of Elisidepsin Treatment Response in Breast and Pancreatic Cancer Cell Lines

**DOI:** 10.1371/journal.pone.0053645

**Published:** 2013-01-08

**Authors:** Cristina Teixidó, Rosó Marés, Miguel Aracil, Santiago Ramón y Cajal, Javier Hernández-Losa

**Affiliations:** 1 Molecular Pathology Group, Vall d’Hebron Research Institute, Universidad Autonoma of Barcelona, Barcelona, Spain; 2 Pharmamar, Madrid, Spain; 3 Pathology Department, Vall d’Hebron University Hospital, Universidad Autonoma of Barcelona, Barcelona, Spain; Vanderbilt University, United States of America

## Abstract

Elisidepsin (elisidepsin trifluoroacetate, Irvalec®, PM02734) is a new synthetic depsipeptide, a result of the PharmaMar Development Program that seeks synthetic products of marine origin-derived compounds. Elisidepsin is a drug with antiproliferative activity in a wide range of tumors. In the present work we studied and characterized the mechanisms associated with sensitivity and resistance to elisidepsin treatment in a broad panel of tumor cell lines from breast and pancreas carcinomas, focusing on different factors involved in epithelial-mesenchymal transition (EMT) and the use of HER family receptors in predicting the *in vitro* drug response. Interestingly, we observed that the basal protein expression levels of EMT markers show a significant correlation with cell viability in response to elisidepsin treatment in a panel of 12 different breast and pancreatic cancer cell lines. In addition, we generated three elisidepsin treatment-resistant cell lines (MCF-7, HPAC and AsPC-1) and analyzed the pattern of expression of different EMT markers in these cells, confirming that acquired resistance to elisidepsin is associated with a switch to the EMT state. Furthermore, a direct correlation between basal HER3 expression and sensitivity to elisidepsin was observed; moreover, modulation of HER3 expression levels in different cancer cell lines alter their sensitivities to the drug, making them more resistant when HER3 expression is downregulated by a HER3-specific short hairpin RNA and more sensitive when the receptor is overexpressed. These results show that HER3 expression is an important marker of sensitivity to elisidepsin treatment.

## Introduction

Elisidepsin (elisidepsin trifluoroacetate, Irvalec®, PM02734), a synthetic cyclic peptide originally isolated from the marine mollusk *Elysia rufescens* [1], is a cytotoxic anticancer agent [2], [3], [4]. Elisidepsin does not exhibit a linear cytotoxic dose-response and acts independently of the multidrug resistant status of various tumor cell lines [5]. The primary mechanisms of action of elisidepsin have not been identified, although multiple cellular targets have been described, many of which, due to the hydrophobic nature of the compound, are associated with the cell membrane [6], [7], [8], [9].

One of the several targets that are proposed to be involved in the cellular response to elisidepsin treatment is the human epidermal growth factor receptor family (HER) with several *in vitro* studies identifying HER3 and the downstream signaling pathway PI3K-AKT as major determinants of the cytotoxic activity of elisidepsin [10], [11]. Moreover, it has recently been postulated that elisidepsin induces the redistribution of HER3 from the plasma membrane to intracellular vesicles without comparable effects on HER1 and HER2, suggesting that it is HER3 that plays a key role in determining sensitivity to the drug [9].

On the other hand, specifically in relation to epithelial cells, one of the best-described processes that affects the composition of the cell membrane is that of the epithelial-mesenchymal transition (EMT), which is where cells downregulate their cell-cell junctions and acquire spindle cell morphology [12], [13]. The EMT plays an important role in development [14], [15], particularly in gastrulation and neural crest migration [14]. A critical component is the loss of type I cadherins that maintain stable cell-cell contacts through adherens junctions and desmosomes [16], [17]. To preserve cellular shape and polarity, the intracellular domains of cadherins connect to the actin cytoskeleton through α-catenin and β-catenin [18], [19], [20].

In most cases, this is associated with transcriptional repression of E-cadherin [21], [22], which in turn increases cell invasiveness [13], [22], [23], [24]. Several specific repressor factors have been identified, such as the zinc-finger domain-containing Snail and Slug factors [25], and the basic helix-loop-helix factor Twist, all of which can bind to the so-called E-boxes within the cadherin-1 (CDH1) gene promoter [25], [26]. Their function is regulated by oncogenic pathways, particularly by AKT, glycogen synthase kinase 3β (GSK-3β), NF-κB, RAS and SRC, some of which have been described as potential elisidepsin targets [15], [27], [28].

In this scenario, until the proposed above targets are validated, robust models that permit the identification novel predictive biomarkers are essential. To this end, and due to the increasing evidence supporting a role for the EMT in the progression of many cancer types, with critical roles in invasion and metastatic dissemination, we decided to study both HER3 and EMT as new predictive markers of elisidepsin treatment sensitivity in a panel of breast and pancreatic cell lines.

In this report, we show that continued exposure to elisidepsin is correlated with a downregulation of epithelial markers in four different cancer cell types (pancreatic, breast, lung and colon). This behavior is further accompanied by several morphological and signaling changes, resulting in the upregulation of mesenchymal markers. Furthermore, we investigated the effect of the drug on the expression of HER proteins and systematically compared the elisidepsin sensitivity of cell lines overexpressing and knocking-down HER3 receptor. Finally, we identified HER3 expression as the most important sensitivity marker of elisidepsin studied.

## Results

### Cancer Cell Line Sensitivity to Elisidepsin

We performed cell viability assays in a panel of 12 cell lines (6 breast cancer cell lines and 6 pancreatic carcinoma cell lines) to determine if there was a correlation between epithelial or mesenchymal expression markers and cell sensitivity to elisidepsin. Cells were treated with increasing concentrations of the compound for 72 h. The half maximal (50%) inhibitory concentration (IC_50_) values for elisidepsin, as measured by a crystal violet assay using a spectrophotometer, ranged from 0.075 to 14 µM within the cell line panel (Fig. 1A).

**Figure 1:** Elisidepsin sensitivity. A) Elisidepsin IC_50_s were determined in a panel of breast (left) and pancreatic (right) cancer cell lines using a crystal violet assay. Cells were exposed to elisidepsin for 72 h. Results are shown as the mean ± SD of at least three independent experiments. B) Cell proliferation in parental and subtoxic elisidepsin-treated cells. Cumulative numbers of cell divisions [shown as population doubling level (PDL)] are shown for MCF-7 and MiaPaCa-2 cells until passage 5. Proliferation of MCF-7 (IC_50_∶0.4 µM) and MiaPaCa-2 (IC_50_∶14 µM) cells was suppressed when elisidepsin was added to the culture at subtoxic doses (0.2 and 1 µM, respectively). The number of MiaPaCa-2 and MCF-7 seeded cells were 1.25×10^5^ and 1.4×10^5^, respectively. Each growth curve was performed at least twice with similar results, SDs are shown, and each time point was performed in duplicate. P, passage.

According to the results of a previous paper from our lab and others [27], [28], only those cells with an IC_50_ value under or equal to 1 µM are considered sensitive to the elisidepsin. MDA-MB-231, PANC-1 and MiaPaCa-2 cell lines were the only cell lines that had an IC_50_ value higher than 1 µM (6.5, 7.5 and 14 µM, respectively). The other cell lines were classed as being sensitive to the drug (with IC_50_ values ranging from 0.075 to 0.6 µM).

The effect of elisidepsin is not considered to be time-dependent as no significant difference in the ratio of IC_50_ values was seen by Sewell et al. [7] following 1 h exposure and continuous exposure. However, when we treated the cells with continuous exposure to a subtoxic dose (i.e. lower than the IC_50_) the cells grew more slowly than the parental ones (Fig. 1B). Recent studies have shown that the potent cytotoxic activity of elisidepsin is exerted very rapidly through insertion of the drug molecule into the plasma membrane, which causes a drastic loss in membrane integrity [8]. However, we found that, despite elisidepsin-induced loss of membrane integrity, those cells that remained alive after treatment could recover and proliferate again (Fig. S1). This was shown by treating MCF-7 cancer cell lines with 1 µM elisidepsin for 4 h, removing the drug and measuring proliferation at different time points. More than 50% of cells died after 4 h drug treatment but when the media was replaced the cells recovered and their viability increased.

### Correlation between EMT Markers and Elisidepsin Cell Sensitivity

In order to evaluate EMT protein expression levels and correlate them with the sensitivity of the cell lines to elisidepsin, we performed different analyses using western blot, immunofluorescence and immunohistochemistry (IHC) in a panel of 12 cell lines. The protein expression of E-cadherin, β-catenin, vimentin, Slug, Snail and Twist-1 were assessed by immunocytochemical and western blot analysis, while the protein expression of E-cadherin, β-catenin, and vimentin were evaluated by immunohistochemical analysis.

We aimed to determine whether the various elisidepsin-sensitive cancer cell lines shared similar basal levels of EMT genes. In the breast cancer cell lines we found E-cadherin expression in the sensitive cell lines. All cell lines had detectable expression of β-catenin, whereas Slug expression was variable and not related to their sensitivity to elisidepsin. Furthermore, Snail expression was only found in MDA-MB-435, and all the cell lines that exhibited levels of Twist-1 and vimentin were less sensitive to the drug (Figs. 2A–C). In contrast, elisidepsin-sensitive pancreatic carcinoma cell lines expressed E-cadherin and β-catenin, whereas the less sensitive cells expressed Slug. Lastly, Snail, Twist-1 and vimentin expression was found in sensitive and insensitive cell lines alike (Figs. 3A–C). To summarize, E-cadherin protein was significantly expressed in the sensitive cell lines independently of their tumoral origin (Mann-Whitney test: p  = 0.0364; Fig. S2), and vimentin was significantly expressed in the less sensitive ones (Mann-Whitney test: p  = 0.0364). On the other hand, Twist-1 and Snail proteins were found in all less sensitive cell lines (Mann Whitney test: p  = 0.0636 and p  = 0.1000, respectively), with the exception of two sensitive cell lines that were positive for vimentin expression (CFPAC and AsPC-1), one sensitive cell line that was positive for Twist-1 expression (CFPAC) and another one that was positive for Snail expression (SKBR3).

**Figure 2:** Expression of EMT markers associated with elisidepsin sensitivity in breast cancer cell lines. Protein expression levels of different EMT markers were evaluated by immunocytochemistry (A), western blot (B) and IHC (C). A) Immunocytochemistry of two epithelial (E-cadherin and β-catenin) and four mesenchymal markers (vimentin, Slug, Snail and Twist). Magnification 100x. B) E-cadherin, β-catenin, Slug, Snail, Twist, vimentin and β-actin (loading control) were detected by western blot analysis using 50 µg of total protein. C) Basal levels of E-cadherin, β-catenin and vimentin were analyzed by IHC. Magnification 20x. Each experiment was performed at least in duplicate.

**Figure 3:** Expression of EMT markers associated with elisidepsin sensitivity in pancreatic cancer cell lines. E-cadherin, β-catenin, vimentin, Slug, Snail and Twist basal expression levels were evaluated by immunocytochemistry (A) and western blot (50 µg of protein/lane) (B). Magnification 100x. Membranes were stripped and reprobed with anti-β-actin as an internal control. C) E-cadherin, β-catenin and vimentin protein expression levels were evaluated by IHC. Magnification 20x. These analyses were performed in duplicate.

### HER3 Expression Levels Correlate with Elisidepsin Cell Sensitivity

The primary mechanisms of action of elisidepsin remain to be elucidated but we and other groups have found that after 4 h treatment with 1 µM elisidepsin, HER3 receptor levels are downregulated in a panel of different cell lines, including lung, breast, melanoma and colon carcinomas [10], [11]. To determine if HER3 protein expression levels correlate with the sensitivity of the cell lines to elisidepsin, we performed IHC (Fig. 4A) and western blot analysis (Fig. 4B) in all cell lines. Cell lines that were less sensitive to elisidepsin had little to no HER3 while sensitive cell lines expressed significantly increased levels of this protein (Mann-Whitney test: p  = 0.0091; Fig. S3). In addition, others members of the HER family were checked by western blot (Fig. 4B) but no correlations with elisidepsin sensitivity were found with HER1, HER2 and HER4 (Mann-Whitney test: p  = 0.7273, p  = 0.5182 and p  = 0.8909, respectively).

**Figure 4:** HER3 expression levels correlate with cell sensitivity to elisidepsin. A) Cell pellets were fixed in formalin, embedded in paraffin and a HER3 IHC was performed. Cell lines more sensitive to elisidepsin had significant HER3 levels. Magnification 40x. B) Basal expression levels of HER family members were analyzed by western blot; an association between HER3 expression and elisidepsin sensitivity was observed (Mann-Whitney test: p  = 0.0091; Fig. S3). Cell lines less sensitive to elisidepsin (MDA-MB-231, PANC-1 and MiaPaCa-2) did not show significant HER3 protein levels, while PANC-1 and MiaPaCa-2 cell lines show levels of other HER family members. No correlation was observed with HER1, HER2 and HER4 expression levels (Fig. S3). These protein expression levels were analyzed in duplicate and 50 µg of protein of cell lysate were loaded in each lane.

### Acquired Resistance to Elisidepsin Induces an EMT Phenotype

Three elisidepsin-resistant cancer cell lines [one breast (MCF-7) and two pancreatic (HPAC, AsPC-1)] were generated by continuous exposure to increasing concentrations of the drug (see Material and Methods). Cancer cell lines were exposed to elisidepsin at a starting concentration of its IC_50_. Elisidepsin concentration was increased every week until cells became resistant to the drug, after approximately 12 months in the case of MCF-7, and after approximately 4 months in the case of HPAC and AsPC-1. The morphology of the resistant cancer cell lines was modified after continuous exposure to the drug when compared to that of the parental cell lines (data not shown). Our hypothesis was that the loss of epithelial markers observed in our panel of cancer cell lines could be responsible for the resistance to elisidepsin treatment, which would in turn result in the acquisition of mesenchymal markers in these cells.

We then performed western blot analysis of the cancer cell lines with acquired resistance and compared them to the corresponding parental control cells. We identified that the three different cancer cell types with acquired resistance to elisidepsin had altered basal levels of EMT markers (Fig. 5A). All resistant cell lines showed decreased E-cadherin, γ-catenin and increased vimentin and Twist-1 expression. β-catenin expression was downregulated in the resistant HPAC and AsPC-1 cancer cell lines but upregulated in the MCF-7. In contrast, levels of Slug and Snail were upregulated in the resistant cancer cell lines HPAC and AsPC-1 but no differences were found in the breast carcinoma MCF-7 cell line.

**Figure 5:** Acquired resistance to elisidepsin induces an EMT phenotype. A) Cells were lysed, proteins were extracted and western blots were performed with equal amounts of cell lysate (50 µg protein). Expression of epithelial (E-cadherin, β-catenin, γ-catenin)- and mesenchymal (vimentin, Slug, Snail, Twist)-associated proteins differentiates between elisidepsin-sensitive and elisidepsin-resistant cell lines. β-actin was used as an internal control. These western blots were performed in triplicate. B) Expression levels of HER1, HER2, HER3, HER4, pAkt, and pMAPK were analyzed by western blot using 50 µg of protein cell lysate. The membranes were stripped and reprobed with anti-β-actin to verify equal protein loading. C, control; R, resistance.

We also performed the same approach in different resistant cell lines from colon and lung (HCT116 and A549, respectively) with similar results (Fig. S4). Analysis by western blot confirmed that acquired resistance to elisidepsin is associated with a switch to the EMT state.

Furthermore, we wanted to see if these cells also showed different expression levels of HER family members and proteins of their signaling pathways. We observed that the levels of all HER family members and their downstream signaling partners were downregulated in all resistant cancer cell lines (Figs. 5B and S4). A suppression of downstream signaling was similarly seen in the breast and pancreatic resistant cell lines, and the same expression pattern was also observed in other colon and lung resistant cell lines, highlighting the relevance of this phenomena.

### Modulation of HER3 Affects Cancer Cell Line Sensitivity to Elisidepsin

Based on previous studies from our group and others demonstrating that elisidepsin downregulates the HER3 receptor tyrosine kinase and that high expression of HER3 is prevalent in a broad number of different tumor cells, we investigated if modulation of protein expression levels of the HER3 receptor affects sensitivity to elisidepsin in a panel of tumor cell lines with variable expression of this receptor.

To examine this experimentally, we utilized a shRNA construct to stably reduce HER3 expression in a panel of cell lines (Fig. 6). Stable clones of HER3 shRNA and LUC shRNA (control) vector-transfected cells were selected and examined for expression of HER3. As expected, levels of HER3 were significantly reduced in HER3-transfected cells, but not in those containing the pLKO LUC shRNA vector alone, indicating that the decrease in HER3 was not due to non-specific effects of introducing shRNA into the cells. Next, cell viability assays were performed to analyze elisidepsin sensitivity in the generated cells. Figure 6 shows that cells that have reduced levels of HER3 due to shRNA-mediated knockdown of its expression showed loss of sensitivity to elisidepsin treatment in comparison to control cell lines.

**Figure 6:** Loss of HER3 expression decreases the sensitivity to elisidepsin treatment. Cell viability after treatment with various concentrations of elisidepsin for 72 h was determined in SKBR3 (A), MCF-7 (B), MDA-MB-231 (C), MDA-MB-435 (D), BT474 (E), BxPC-3 (F), HPAC (G) and AsPC-1 (H) cells. HER3 expression was downregulated with shRNA (grey squares); LUC shRNA transfected cells were used as the control (black diamonds). Mean, SD, and IC_50_ values are shown from three independent experiments. Cell viability was measured using a crystal violet assay. Before performing the viability experiments, all cell lines were checked by western blot using 50 µg of protein to confirm their levels of HER3 expression.

To investigate whether ectopic HER3 expression affects the elisidepsin sensitivity of low HER3-expressing cells, the levels of HER3 were increased by transfecting cells with a cDNA encoding HER3, which resulted in increased sensitivity of the cells to elisidepsin. In comparison to control cells transfected with a LUC vector, decreased cell viability was noted in HER3-transfected cells (Fig. 7). Altogether, these results suggest that ectopic HER3 expression sensitizes these cells to elisidepsin treatment.

**Figure 7:** Upregulation of HER3 increases elisidepsin sensitivity. Cell viability after treatment with various concentrations of elisidepsin for 72 h was determined in PANC-1 (A), MiaPaCa-2 (B), MDA-MB-435 (C) and MDA-MB-231 (D) cells. Stable cell lines with an upregulation of HER3 expression (with the pIRES HER3) are shown with white circles while black diamonds are used for LUC-transfected control cells (with the pIRES-LUC). Mean, SD, and IC_50_ values are shown from three independent experiments. Cell viability was measured by a crystal violet assay. Before performing the viability experiments, all cell lines were checked by western blot using 50 µg of protein to confirm their levels of HER3 expression.

## Discussion

Elisidepsin is a novel marine compound with a potent cytotoxic activity in various tumor cell lines. The mechanisms of actions of this compound remain poorly understood, although several targets have been proposed to be involved in the cellular response to elisidepsin treatment, such as fatty acid-containing ceramides, fatty acid 2-hydroxylase (FA2H), lysosomes, lipid rafts and epithelial growth factor receptors, including the HER receptors [10], [29], [30], [31], [32], [33].

In the present study we explored whether basal levels of EMT markers and HER receptor proteins could be predictive markers for elisidepsin treatment. The role of the cell membrane as an important target of elisidepsin was studied in breast and pancreas cancer cell lines. Basal levels of EMT protein expression markers showed a significant correlation with the cell viability response to elisidepsin treatment in a panel of 12 different cancer cell lines. The epithelial marker E-cadherin protein was significantly expressed in the sensitive cell lines (p  = 0.0364) while expression of the mesenchymal markers vimentin, Twist-1 and Snail, was found in all cell lines with reduced sensitivity to the drug.

Furthermore, this study showed that continuous exposure to elisidepsin correlates with a downregulation of epithelial markers in 4 different cancer cell types (breast, pancreas, lung and colon). Loss of epithelial markers was further evidenced by the detection of morphological changes in the cells. These changes, which were observed after continuous long-term exposure of different cell types to elisidepsin, suggest that the drug is able to modify the composition of the plasma membrane. This behavior was further accompanied by signaling changes, resulting in the upregulation of mesenchymal markers. This analysis confirmed that acquired resistance to elisidepsin is associated with a switch to the EMT state.

On the other hand, regarding HER family receptors, we observed an association between HER3 protein expression and sensitivity to elisidepsin treatment in a variety of cell lines (p  = 0.0091). The other members of the HER family were also checked by western blotting and we did not find any significant correlation. Interestingly, HER4 expression was observed in 4 out of 5 elisidepsin-sensitive breast cancer cell lines, and further studies that include more breast cancer cell lines are necessary to establish the potential predictive marker of the HERs for elisidepsin sensitivity in breast cancer models. Cell lines that were less sensitive to elisidepsin had lower or undetectable levels of HER3 in comparison with sensitive cell lines, supporting a hypothetical role for HER3 in the cellular response to this drug, although other authors propose that HER3 is part of a secondary process involving cell membrane alterations due to elisidepsin treatment [9] or to a reduction in the proliferation rate in those cells with less HER3 expression. Importantly, we could not discard the possibility that elisidepsin may affect other signaling pathways, such as those of the transforming growth factor-β (TGF-β) family, which potentially plays a role in both EMT and HER3 expression.

Malignant cells commonly possess overactive signal transduction cascades that provide potential selective targets for antitumor drugs [34]. Based on previous studies in which we observed elisidepsin treatment-induced HER3 downregulation [11], in addition to the fact that high expression of the HER3 receptor tyrosine kinase is prevalent in tumor cells, including cancers of the breast, ovary and prostate [35], [36], [37], [38], [39], [40], [41], [42], we correlated basal protein expression levels of HER3 with sensitivity to elisidepsin in a panel of tumor cell lines with variable expression of this receptor and found that downregulation of HER3 exerted a protective effect against elisidepsin cytotoxicity. In fact, HER3 significantly increases cell sensitivity in all cell lines studied, supporting previous indications that HER3 could be a good predictive marker of cell sensitivity to elisidepsin.

In summary, we present solid evidence that sensitivity to elisidepsin correlates with HER3 receptor expression. However, it remains to be elucidated why elisidepsin affects HER3 and why its effects depend on HER3 expression.

## Materials and Methods

### Chemicals

Elisidepsin (Figure S5) was obtained from PharmaMar (Madrid, Spain) as a lyophilized powder. It was reconstituted in dimethyl sulfoxide (DMSO; Sigma-Aldrich, Taufkirchen, Germany)/ethanol (1∶1) as a 1 mM stock solution, which was stored in aliquots at −20°C. Drug dilutions were freshly prepared before each experiment in order to avoid degradation.

### Cells and Cell Culture

Cell lines were obtained from the American Type Culture Collection (VA, USA). The following cell lines were maintained in RPMI 1640 with 4 mM L-glutamine: MDA-MB-435, MDA-MB-231, MCF-7 and SKBR3 (breast carcinoma), and AsPC-1 and BxPC-3 (pancreas carcinoma). The following cell lines were maintained in Dulbecco's modified Eagle's medium (DMEM) with 4 mM L-glutamine and 4.5 g/L glucose: HCT116 (colon carcinoma), MDA-MB-468 (breast carcinoma), and HPAC, PANC-1 and MiaPaCa-2 (pancreas carcinoma). A549 (lung carcinoma) was maintained in Ham's F-12 medium supplemented with 1 mM L-glutamine. Finally, DMEM:Ham's F12 (1∶1 mixture) supplemented with 1 mM L-glutamine was used to maintain BT474 (breast carcinoma). HPAC resistant to elisidepsin 8 µM and AsPC-1 resistant to elisidepsin 4.5 µM were generated by continuous exposure to the drug for ∼4 months, while HCT 116 resistant to elisidepsin 100 µM, A549 resistant to elisidepsin 25 µM, and MCF-7 resistant to elisidepsin 4 µM were generated by continuous exposure to the drug for ∼1 year. The media for all cell lines were supplemented with 10% fetal bovine serum, 100 U/mL penicillin, 100 µg/mL streptomycin and 10 mM HEPES and were cultured in a 37°C humidified atmosphere containing 95% air and 5% CO_2_.

### Western Blots

Immediately prior to use in western blotting, cultured cells were lysed and collected in lysis buffer. Lysates were centrifuged and supernatants were collected for protein concentration determination using the Bradford (Bio-Rad Protein Assay, Munich, Germany) method. Equal amounts of protein were separated by 8% sodium dodecyl sulfate (SDS)-polyacrylamide gel electrophoresis (PAGE) gels, electrophoresed at 100 V and electroblotted onto polyvinylidene difluoride membranes (Merck Millipore, Billerica, MA) at 0.4 A at room temperature. Blots were blocked in 5% nonfat dry milk in phosphate-buffered saline (PBS) for 1 h at room temperature. After blocking, membranes were incubated overnight with primary antibodies against HER1 (F4, Sigma-Aldrich); HER2 (CB11, BioGenex, Fremont, CA, USA); HER3 (2F12, NeoMarkers, Fremont, CA); HER4 (111B2), Akt (#9272), γ-catenin (#2309) and Snail (L70G2; all from Cell Signaling, Beverly, MA, USA); MAPK (C-14), Slug (H-140) and Twist-1 (H-81; all from Santa Cruz, Heidelberg, Germany); β-actin (A2228, Sigma-Aldrich); vimentin (V9, Dako, Sant Just Desvern, Spain); and E-cadherin and β-catenin (Novocastra, Badalona, Spain). After incubation with horseradish peroxidase-conjugated secondary antibodies, antigen-antibody complexes were visualized using enhanced chemiluminescence (Amersham Biosciences, Dreieich, Germany). Western blots were repeated in independent conditions at least twice and representative blots are shown. Densitometrical quantification of autoradiograms was performed using ImageJ software (version 1.41o, National Institutes of Health, Bethesda, MD) by normalizing to the intensity of β-actin in each sample and are expressed in arbitrary densitometric units.

### Immunocytochemistry

Cells were seeded on coverslips at 60% confluence, fixed in 4% formaldehyde/PBS, permeabilized in 100% methanol for 20 min, and blocked in 2% BSA for 1 h. Fixed cells were incubated with anti-E-cadherin (clone 36B5, 1∶50) and anti-β-catenin (Novocastra, 1∶50), anti-Snail (Cell Signaling, 1∶50), anti-Vimentin (Dako, 1∶50), and anti-Slug and anti-Twist-1 (Santa Cruz, 1∶50) overnight at 4°C. After washing with PBS, cells were incubated for 1 h in blocking buffer at room temperature with either 1∶800 Alexa Fluor 546 rabbit anti-mouse IgG (Invitrogen, Barcelona, Spain) or 1∶200 Alexa Fluor 647 mouse anti-human (Invitrogen). Cells were washed twice with PBS and once with distilled water. Finally, cells were mounted in Citifluor (Leicester, UK) before observation and analysis with fluorescence microscopy.

### Immunohistochemical Staining

IHC using the avidin-biotin-peroxidase technique was performed for each antibody. Five-micron-thick sections were cut from formalin-fixed, paraffin-embedded cell pellets and placed on poly-L-lysine-coated glass slides. Sections were deparaffinized in xylene and rehydrated in graded alcohol. Endogenous peroxidase was blocked by immersing the sections in 0.1% hydrogen peroxidase in absolute methanol for 20 min. For antigen retrieval, the tissue sections were heated in a pressure cooker in 10 mM citric acid monohydrate, pH 6.0, for 5 min, and then incubated with primary antibodies for 60 min at room temperature. IHC was performed with the Benchmark XT slide stainer (Ventana Medical Systems, Inc, Tucson, AZ, USA). The primary antibodies and dilutions used were: anti-HER3 [generated by Dr. Pandiella (IBMCC, Salamanca, Spain), 1∶75], anti-E-cadherin (Dako, pre-diluted), anti-β-catenin (Novocastra, 1∶50) and anti-vimentin (Dako, pre-diluted). All slides were hematoxylin counterstained, dehydrated, and mounted. Negative controls were performed by omitting the primary antibody and showed minimal non-specific signal.

### Cell Growth Assay

Cells were plated overnight at a density of 50,000 cells/well. Cell lines were treated with various concentrations of elisidepsin for 72 h. At least 3 wells were used for each condition and cell viability was measured by a crystal violet assay. Briefly, cells were fixed after each treatment in 1% glutaraldehyde for 20 min, washed twice in PBS, stained with 0.1% crystal violet for 30 min and then washed with abundant deionized water. Colorant was recovered using 5% acetic acid and optical density was measured at 590 nM with an ELISA plate reader.

### Plasmids and Cell Transfection

The pIRES-HER3 and the pIRES-Luciferase (LUC) were kindly donated by Dr. Scaltriti (Vall d’Hebron University Hospital Research Institute, Barcelona, Spain). The pIRES-LUC was used as a control for transfection. The pIRES vectors confer hygromycin resistance. Cells were transfected for 12 h with Jet Pei (Polyplus-Transfection, Illkirch, France). To eliminate untransfected cells and generate stably expressing HER3 cell lines, medium supplemented with hygromycin (Sigma-Aldrich) was added 24 h after transfection, and cells underwent selection for 10 days.

### Lentivirus shRNA Production and Transduction

Short hairpin RNAs (shRNAs) were used for inhibiting HER3 expression in different cancer cell lines. The following sequences were used: shHER3_3.1F: GATCCAAGAGCGACTAGACATCAAGCTTCAAGAGAGCTTGATGTCTAGTCCCTCTTTTTTTACGCGTG, shHER3_3.1R: AATTCACGCGTAAAAAAAAGAGCGACTAGACATCAAGCTCTCTTGAAGCTTGATGTCTAGTCGCTCTTG; shHER3_3.3F: ATCCGCCAATACCAGACTGTACTTCAAGAGAAGTACAGTGTCTGGTATTGGTTTTTTACGCGTG, and shHER3_3.3R: AATTCACGCGTAAAAAACCAATAC CAGACACTGTACTCTCTTGAAGTACAGTGTCTGGTATTGGCG. The different sequences were cloned into the lentiviral vector pLKO.1 (Sigma-Aldrich). The pLKO.1-shRNA LUC was used as a control for transfection. All vectors encode puromycin resistance. Plasmids pVSVG and pCMVΔR8.91 for the expression of packaging and envelope proteins were kindly provided by Dr. Peeper (VU University Medical Center, Amsterdam, The Netherlands). Two plates seeded with 1.5×10^6^ HEK 293T cells were co-transfected in DMEM 10% FBS with 2 µg of pLKO.1, 2 µg of pCMVΔR8.91 and 2 µg of pVSVG and incubated overnight. Cells were washed and incubated in 10% CO_2_ with medium containing 5% FBS. After 48 h, the virus-containing supernatant was recovered and filtered with 0.45 nM filters (Sarstedt, Nümbrecht, Germany).

Titration was performed by infecting cells with the recovered viral particles in the presence of 4 µg/mL polybrene (Sigma-Aldrich). Western blot was used to assess the silencing efficacy of the two shHER3 sequences, and the most effective one (shHER3.3) was chosen. To obtain cell lines with stable depletion of HER3, infected cells were selected with puromycin for three days.

### Statistical Analysis

Statistical studies were performed with the Statistical Package for the Social Sciences (SPSS 15.0; SPSS, Chicago, IL). The Mann-Whitney test was used to find associations of the parameters analyzed between two previously selected groups, Sensitive (includes cell lines with an elisidepsin IC_50_≤1 µM) and Less Sensitive (includes cell lines with an elisidepsin IC_50_>1 µM). Cell growth data are expressed as the mean ± standard deviation (SD). Statistical significance was set at a two-tailed p value of 0.05.

## Supporting Information

Figure S1 **MCF-7 cells can recover after elisidepsin treatment.** A) Cells were treated with 1 µM of elisidepsin for 4 h, the culture medium was changed and cells were maintained in the fresh medium for 4, 24, 48 and 72 h. HER1-4 protein expression levels were analyzed by western blot using 50 µg of protein from total MCF-7 cell lysates loaded in SDS-PAGE gels. Membranes were stripped and reprobed with anti-β-actin to verify equal protein loading. B) Cells were treated with 1 µM of elisidepsin for 4 h and proliferation was measured by a crystal violet assay at different time points (white squares) and compared to untreated cells (black diamonds). Results are expressed as the mean ± SD of two independent experiments. C, control.
(TIF)

Figure S2 **Statistical analysis of EMT basal expression levels of breast and pancreas cancer cell lines.** Levels of ErbB3 protein were quantified using western blot analysis (see Material and Methods) by densitometry. The graph represents the relative ErbB3 expression in elisidepsin-sensitive (IC_50_≤1 µM) and -resistant (IC_50_>1 µM) cell lines. The Mann-Whitney test showed a statistically significant p value of 0.015.
(TIF)

Figure S3 **Elisidepsin cell sensitivity is associated with HER3 expression levels.** Levels of HER1, HER2, HER3 and HER4 protein were quantified with western blot analysis (Fig. 4) and subsequent densitometry. Cells that have an elisidepsin IC_50_ value of ≤1 µM were considered sensitive to the drug. The graph represents the HER family members expression relative to elisidepsin sensitivity. A statistically significance relationship between HER3 expression levels and elisidepsin sensitivity was found (Mann-Whitney test: p  = 0.0091) but not with the other members.
(TIF)

Figure S4 **Generation and characterization of elisidepsin-resistant cell lines from colon and lung.** A) Cells were lysed, proteins were extracted and western blots performed with an equal amount of cell lysate (50 µg protein). Expression of epithelial (E-cadherin, β-catenin, γ-catenin)- and mesenchymal (vimentin, Slug, Snail, Twist)-associated proteins differentiates between elisidepsin-sensitive and elisidepsin-resistant cell lines. β-actin was used as an internal control. These western blots were performed in triplicate. B) Expression levels HER1, HER2, HER3, HER4, pAkt, and pMAPK were analyzed by western blot using 50 µg of protein cell lysate. The membranes were stripped and reprobed with anti-β-actin to verify equal protein loading. HCT 116 (C) and A549 (D) elisidepsin-sensitive cancer cell lines were rendered resistant by persistent exposure to increasing concentrations of elisidepsin. Cells were treated with elisidepsin at the indicated concentrations for 72 h and cell viability was measured using a crystal violet assay. Error bars show the SD of three replicate experiments. C, control; R, resistance.
(TIF)

Figure S5 **Chemical structure of elisidepsin.**
(TIF)
